The article "Macular Edema and Visual Acuity Observation after Cataract Surgery in Patients with Diabetic Retinopathy" was published in 2022. Journal: J Healthc Eng.

# Macular Edema and Visual Acuity Observation after Cataract Surgery in Patients with Diabetic Retinopathy

**DOI:** 10.1155/2022/3311751

**Published:** 2022-01-25

**Authors:** Ruiying Song, Jing Jiang, Hong Wang

**Affiliations:** Department of Ophthalmology, Yantai Yuhuangding Hospital, Yantai 264000, Shandong Province, China

## Abstract

**Objective:**

The purpose was to explore the effect of cataract surgery on postoperative macular edema and visual acuity in patients with diabetic retinopathy.

**Methods:**

88 patients with diabetic retinopathy treated in our hospital (December 2019–December 2020) were chosen as research subjects and divided into experimental group of 44 patients (52 eyes) and control group of 44 patients (54 eyes) according to the odd and even admission numbers. The control group received laser photocoagulation treatment, while the experimental group underwent cataract surgery. The central macular thickness (CMT) and visual acuity of the two groups after treatment were detected to evaluate the therapeutic effect of different treatment methods on diabetic retinopathy.

**Results:**

No obvious differences in sex ratio, average age, average course of disease, average weight, average BMI, average glycosylated hemoglobin, and residence were found between the two groups (*P* > 0.05). The total clinical effective rate in the experimental group was obviously higher compared with the control group (*P* < 0.05). The CMT at T1, T2, and T3 in the experimental group was obviously lower compared with the control group (*P* < 0.05). The BCVA in the experimental group at 1 month and 3 months after treatment was obviously higher compared with the control group (*P* < 0.05). The VEGF levels of both groups after treatment were obviously lower (*P* < 0.001), and the VEGF level in the experimental group after treatment was obviously lower compared with the control group (*P* < 0.001). The total incidence of complications in the experimental group was obviously lower compared with the control group (*P* < 0.05).

**Conclusion:**

Cataract surgery is a reliable method to improve visual acuity and reduce serum inflammatory indicators in patients with diabetic retinopathy, with better clinical effect than laser photocoagulation, which is recommended for the treatment of diabetic retinopathy.

## 1. Introduction

Macular edema refers to edema caused by fluid infiltration or inflammation in the macular area of the retina, the most sensitive part of the fundus to light, which is an important cause of visual deterioration [1, 2]. Diabetes mellitus is a chronic metabolic disease, and long-term hyperglycemia in the body will lead to ocular microvascular damage, leading to diabetic retinopathy. With the development of the disease, retinal ischemia and hypoxia can increase vascular permeability and eventually lead to diabetic macular edema (DME) [3, 4]. Xueshuantong capsule is a commonly used drug for the treatment of diabetic retinopathy. However, after its administration, nervous system symptoms such as shortness of breath and chest tightness occur, with gastrointestinal side effects in some patients, which seriously affect the therapeutic effect. At present, cataract surgery is the best method to treat diabetic retinopathy, in which the vision of patients is improved by removing the clouded lens and implanting intraocular lens. This treatment method had the advantages of a small incision, less tissue damage, and quick recovery after surgery, which has been confirmed in diseases such as hard nucleus cataract and diabetic retinopathy [5]. However, a study [6] has shown that patients with diabetic retinopathy will have macular thickening and higher possibility of macular edema after surgery. As an adrenocorticotropic hormone, triamcinolone acetonide has vasoconstriction and anti-inflammatory effects. It has been clinically confirmed that intravitreous injection of triamcinolone acetonide in such patients can effectively reduce the incidence of postoperative macular edema, which is of great significance in improving the treatment effect and vision [7, 8]. Based on this, this study aims to explore the effect of cataract surgery on patients with diabetic retinopathy, as well as the effect on macular edema and visual acuity after surgery, summarized and reported as follows.

## 2. Materials and Methods

### 2.1. General Information

88 patients with diabetic retinopathy treated in our hospital (December 2019–December 2020) were chosen as research subjects and divided into experimental group of 44 patients (52 eyes) and control group of 44 patients (54 eyes) according to the odd and even admission numbers. The study was conducted in accordance with the Declaration of Helsinki (as revised in 2013) [9].

### 2.2. Inclusion Criteria

(1) The patients met the diagnostic criteria of fundus lesions and diabetes, namely, symptoms such as excessive drinking, urine, and eating, weight loss, fasting plasma glucose level ≥7.0 mmol/L, and random blood glucose level ≥11.1 mmol/L after fluorescence fundus angiography (FFA) examination; (2) the clinical symptoms included mild blurred vision, retinal hemorrhage, and vitreous hemorrhage; (3) the patients were less than 70 years old; and (4) the patients had indications of cataract surgery, including severe lenticular opacity, poor visual contrast sensitivity, no intraocular infection, and no coagulation disorders.

### 2.3. Exclusion Criteria

(1) The patients were complicated with ocular infection; (2) the patients previously had uveitis, glaucoma, and other intraocular diseases; (3) the patients had received eye surgery; (4) the patients had congenital ocular lesions or ocular lesions caused by radiation and drugs.

### 2.4. Methods

The control group received laser photocoagulation treatment, with compound tropicamide eye drops (SFDA approval no. J20180051; manufacturer: Santen Pharmaceutical Co., Ltd.; specification: 10 ml) to fully dilate their pupils, Alcon eye drops (approval number: H20090082; manufacturer: S.A. Alcon-Couvreur N.V.; specification: 15 ml: 75 mg) for surface anesthesia, and VISULAS 532s laser therapy apparatus (agent manufacturer: Shanghai Huanxi Medical Device Co., Ltd.) for laser photocoagulation. The parameters included a spot diameter of 50–100 *μ*m, power of 200 mW, and exposure time of 0.1 s.

The experimental group received cataract surgery. The blood glucose level was controlled within a reasonable range before surgery. The patients were treated with phacoemulsification combined with intraocular lens implantation by using the American ALCON-infiniti-VI phacoemulsification apparatus. The main incision (a length of about 2.7 mm) was made in the transparent cornea in the temporal side of the eyes, and the continuous circular capsulorhexis was performed. After removing the residual cortex, the multifocal intraocular lens (SA60 D3 type) was implanted. At the end of the surgery, 4 mg of triamcinolone acetonide (SFDA approval no. H53021604; manufacturer: Kunming Jida Pharmaceutical Co., Ltd.; specification: 1 ml: 40 mg) was injected into the vitreous cavity at 3.5 mm behind the corneal limbus. After surgery, the patients received prednisolone acetate eye drops (approval number: H20171243; manufacturer: Allergan Pharmaceuticals Ireland; specification: 5.0 g/L), 3 times/d for 3 consecutive weeks.

### 2.5. Observation Indexes

Efficacy evaluation: after treatment, visual acuity showed improvement of more than 2 lines, and fundus hemorrhage or exudation was significantly improved, which was markedly effective; visual acuity showed improvement of 1-2 lines, and fundus hemorrhage or exudation was improved, which was effective; visual acuity was not improved, and fundus hemorrhage or exudation was not relieved or even aggravated, which was ineffective. Total effective rate = markedly effective rate + effective rate.

Optical coherence tomography (OCT) was used to detect the CMT of both groups before treatment (T0), 1 month after treatment (T1), 2 months after treatment (T2), and 3 months after treatment (T3).

The standard visual acuity chart was used to examine the best corrected visual acuity (BCVA) of both groups before treatment, 1 month after treatment, and 3 months after treatment, and the results were converted to logarithm of the minimum angle of resolution (logMAR).

5 ml of fasting venous blood in both groups was collected before and after treatment, and serum was collected after centrifugation. Enzyme-linked immunosorbent assay (ELISA) was used to determine the vascular endothelial growth factor (VEGF) levels in serum samples. The kits were purchased from Wuhan Adanti Biotechnology Co., Ltd., and operated strictly according to the kit instructions.

The incidence of clinical complications was recorded and compared, including posterior capsule rupture, corneal hydrops, and descemet membrane detachment.

### 2.6. Statistical Methods

All the experimental data were statistically analyzed and processed by SPSS21.0 software and were graphed by GraphPad Prism 7 (GraphPad Software, San Diego, USA). The count data were tested by *X*^2^, expressed by *n*(%), and the measurement data were measured by *t*-test, expressed by ‾*x* ± *s*. The difference was statistically significant when *p* < 0.05.

## 3. Results

### 3.1. Comparison of Clinical Data

No obvious differences in sex ratio, average age, average course of disease, average weight, average BMI, average glycosylated hemoglobin, and residence were found between the two groups (*P* > 0.05), indicating comparability (Table 1).

### 3.2. Comparison of Clinical Efficacy

The total clinical effective rate in the experimental group was obviously higher compared with the control group (*P* < 0.05; Table 2).

### 3.3. Comparison of CMT at Different Time

With no obvious difference in the CMT at T0 between the two groups (*P* > 0.05), the CMT at T1, T2, and T3 in the experimental group was obviously lower compared with the control group (*P* < 0.05; Figure 1).

### 3.4. Comparison of BCVA at Different Time

With no obvious difference in the BCVA before treatment between the two groups (*P* > 0.05), the BCVA in the experimental group at 1 month and 3 months after treatment was obviously higher compared with the control group (*P* < 0.05; Table 3).

### 3.5. Comparison of Serum VEGF Levels

The VEGF levels of both groups after treatment were obviously lower (*P* < 0.05), and the VEGF level in the experimental group after treatment was obviously lower compared with the control group (*P* < 0.05; Figure 2).

### 3.6. Comparison of Complications

The total incidence of complications in the experimental group was obviously lower compared with the control group (*P* < 0.05; Table 4).

## 4. Discussion

Cataract surgery is widely used in clinical treatment. In this surgery, the turbid lens nucleus is broken into chyle by inserting an ultrasonic probe into the small incision in the affected eye's cornea or sclera. The chyle is sucked out by the suction-perfusion system, the lens cortex is sucked out, and the viscoelastic agent is injected. Finally, the intraocular lens is implanted. This surgery has the advantages of short operation time, convenient operation, and small damage to the eye. Clinical investigations [10] show that macular edema is common after cataract surgery, with an incidence rate of 7%–18% and a morbidity peak mostly in 6–9 weeks after surgery. The pathological mechanism is that the liquid infiltration and inflammatory reaction in the macular area of the fundus result in edema, leading to central retinal vein occlusion and retinopathy [11–13]. Some scholars believe that diabetes is a risk factor affecting macular edema. Due to the blood glucose metabolic disorders in patients with diabetic retinopathy, retinal microcirculation and retinal vascular permeability are changed. After cataract surgery, macula is significantly thickened and the risk of macular edema is significantly increased [14–16]. Laser is an important method to treat eye diseases with the advantages of stable wavelength and accurate direction. Different wavelengths to treat various tissues of patients' eyeballs can achieve good therapeutic effect. At the same time, laser treatment can not only consolidate the visual acuity of patients but also greatly reduce complications. Therefore, laser photocoagulation has become a common way to treat diabetic retinopathy, which can effectively occlude the leaky vessels in the macular area and reduce macular edema by water reflux through osmotic pressure, thereby alleviating retinal hypoxia and inhibiting angiogenesis [17–19]. However, the curative effect of laser treatment alone is gradually reduced with time and is difficult to last, so it is of great significance to explore treatment methods with strong and lasting effect. Studies have found that triamcinolone acetonide, as a glucocorticoid, reduces extracellular fluid exudation and inhibits fibroblast proliferation, thereby controlling and alleviating intraocular inflammation in patients [20–22]. Foreign scholars believe that intravitreous injection of triamcinolone acetonide can maintain a high concentration of the drug in the eye for a long time, which is conducive to the exertion of drug efficacy, effectively inhibit the formation of retinal, choroidal, and iris neovascularization, and also be used to treat macular edema caused by various causes [23, 24].

In this study, patients with diabetic retinopathy were treated with laser photocoagulation therapy and cataract surgery respectively, and CMT at T1, T2, and T3 in the experimental group was obviously lower compared with the control group (*P* < 0.05), indicating that cataract surgery obviously reduces CMT of patients and facilitates the improvement of their vision. In addition, VEGF is a glycoprotein against heat and acid, with a highly conserved structure. Immunohistochemical location has found that VEGF can bind to vesicles in endothelial cells, form some holes on the cell membrane that allow passage of biomacromolecules, and promote the transmembrane transport of biomolecules, thereby increasing vascular permeability. This study showed that the VEGF levels of both groups after treatment were obviously lower (*P* < 0.05), and the VEGF level in the experimental group after treatment was obviously lower compared with the control group (*P* < 0.05). VERMA et al. [25] found in their study that the VEGF level of patients with diabetic retinopathy after cataract phacoemulsification of 58.24 ± 7.11 pg/mL was obviously lower than 116.83 ± 6.25 pg/mL of the routine treatment group, indicating that cataract surgery can obviously reduce the VEGF level of patients with diabetic retinopathy, thereby inhibiting the proliferation of endothelial cells and angiogenesis and improving the therapeutic effect. The study has some limitations, such as a small sample size and short follow-up observation time. Therefore, in future studies, the sample size should be further expanded, and the observation time should be extended. In addition, comprehensive visual quality indicators such as color vision and visual field should be added to provide more clinical evidence for the treatment of patients.

In conclusion, cataract surgery is a reliable method to improve visual acuity and reduce CMT in patients with diabetic retinopathy, with high safety. Therefore, its further research will help to provide a better solution for such patients.

## Figures and Tables

**Figure 1:** Comparison of CMT at different time (‾*x* ± *s*). Note: the abscissa represented T0, T1, T2 and T3, and the ordinate represented CMT values (*μ*m). The CMT values at T0, T1, T2, and T3 in experimental group were 429.35 ± 76.45 *μ*m, 366.27 ± 60.35 *μ*m, 332.47 ± 51.62 *μ*m, and 236.62 ± 35.42 *μ*m, respectively. The CMT values at T0, T1, T2, and T3 in the control group were 429.39 ± 76.42 *μ*m, 401.13 ± 58.69 *μ*m, 376.23 ± 51.43 *μ*m, and 271.74 ± 32.17 *μ*m, respectively. ^*∗*^ indicates an obvious difference in CMT values at T1 between the two groups (*t* = 3.015, *P* < 0.05). ^*∗∗*^ indicates an obvious difference in CMT values at T2 between the two groups (*t* = 4.371, *P* < 0.001). ^*∗∗∗*^ indicates an obvious difference in CMT values at T3 between the two groups (*t* = 5.597, *P* < 0.001).

**Figure 2:** Comparison of serum VEGF levels (‾*x* ± *s*). Note: the abscissa represented before and after treatment, and the ordinate represented the VEGF level (pg/mL). The VEGF levels in the experimental group before and after treatment were 208.73 ± 24.65 pg/mL and 57.46 ± 6.94 pg/mL, respectively. The VEGF levels in control group before and after treatment were 208.69 ± 24.69 pg/mL and 118.23 ± 6.68 pg/mL, respectively. ^*∗*^ indicates an obvious difference in VEGF levels of the experimental group before and after treatment (*t* = 39.183, *P* < 0.001). ^*∗∗*^ indicates an obvious difference in VEGF levels of control group before and after treatment (*t* = 23.460, *P* < 0.001). ^*∗∗∗*^ indicates an obvious difference in VEGF levels between the two groups after treatment (*t* = 41.848, *P* < 0.001).

**Table 1:** Comparison of clinical data.

Items	Experimental group (*n* = 44)	Control group (*n* = 44)	*χ* ^2^/*t*	*P*
Gender			0.046	0.831
Male	23 (52.27%)	24 (54.55%)		
Female	21 (47.73%)	20 (45.45%)		
Average age (years old)	56.72 ± 6.58	56.69 ± 6.54	0.021	0.983
Average course of disease (year)	2.46 ± 1.36	2.48 ± 1.41	0.068	0.946
Average weight(kg)	72.62 ± 3.41	72.59 ± 3.44	0.041	0.967
Average BMI (kg/m^2^)	21.32 ± 1.22	21.36 ± 1.25	0.152	0.880
Average glycosylated hemoglobin (%)	6.53 ± 0.34	6.58 ± 0.36	0.670	0.505
Residence			0.046	0.831
Urban area	20 (45.45%)	21 (47.73%)		
Rural area	24 (54.55%)	23 (52.27%)		

**Table 2:** Comparison of clinical efficacy (*n* (%)).

Group	*n*	Markedly effective	Effective	Ineffective	Total effective rate
Experimental group	52	23(44.23%)	25(48.08%)	4(7.69%)	92.31%(48/52)
Control group	54	17(31.48%)	25(46.30%)	12(22.22%)	77.78%(42/54)
*X* ^2^					4.364
*P*					< 0.05

**Table 3:** Comparison of BCVA at different time (‾*x* ± *s*).

Group	*N*	Before treatment	1 month after treatment	3 months after treatment
Experimental group	52	0.29 ± 0.15	0.77 ± 0.23	0.79 ± 0.21
Control group	54	0.30 ± 0.13	0.62 ± 0.26	0.65 ± 0.23
t		0.367	3.142	3.269
*P*		0.714	<0.05	<0.05

**Table 4:** Comparison of complications (*n*(%)).

Group	*n*	Posterior capsule rupture	Corneal edema	Aqueous capsule avulsion	Total incidence
Experimental group	52	1(1.92%)	1(1.92%)	0(0.00%)	3.85%(2/52)
Control group	54	2(3.70%)	4(7.41%)	3(5.56%)	16.67%(9/54)
*X* ^2^					4.682
*P*					<0.05

## Data Availability

Data to support the findings of this study are available upon reasonable request from the corresponding author.
